# Effect of Root Canal Therapy Combined with Full Crown Restoration on the Level of Inflammatory Factors and Chewing Function in Patients with Cracked Teeth and Chronic Pulpitis

**DOI:** 10.1155/2021/3299349

**Published:** 2021-08-30

**Authors:** Ying Lu, Ning Wu, Bin Ma, Feng Qin

**Affiliations:** ^1^Department of Stomatology, Shidong Hospital of Yangpu District, Shanghai 200438, China; ^2^Department of Stomatology, Liqun Hospital of Putuo District, Shanghai 200333, China; ^3^Department of Endodontics, Shanghai Ninth People's Hospital, Shanghai Jiao Tong University School of Medicine, Huangpu, Shanghai 200011, China; ^4^National Clinical Research Center for Oral Diseases Huangpu District, Shanghai 200011, China; ^5^Shanghai Key Laboratory of Stomatology & Shanghai Research Institute of Stomatology, Huangpu, Shanghai 200011, China

## Abstract

**Objective:**

To explore the clinical effect of root canal therapy combined with full crown restoration in patients with cracked teeth and chronic pulpitis.

**Methods:**

From May 2018 to June 2020, 87 patients with cracked teeth and chronic pulpitis in our hospital were selected; the patients were randomly divided into the control group and the research group by random number method. The control group only used root canal therapy; the research group used root canal therapy combined with full crown restoration. The therapeutic effect, levels of inflammatory factors, chewing function, periodontal index, complications, and quality of life were compared between the two groups.

**Results:**

The total effective rate of the research group (97.78%) was better than the total effective rate of the control group (85.71%) (*P* < 0.05). Compared with before treatment, the serum levels of interleukin-1*β* (IL-1*β*), IL-6, and C-reactive protein (CRP) of the two groups of patients decreased after treatment. After treatment, compared with the control group, the serum levels of IL-1*β*, IL-6, and CRP in the research group decreased (*P* < 0.05). Compared with before treatment, the bite force of teeth and chewing efficiency of the two groups of patients increased after treatment. After treatment, compared with the control group, the bite force of teeth and chewing efficiency of the research group increased (*P* < 0.05). Compared with before treatment, the plaque index (PLI), probing depth (PD), gingival sulcus bleeding index (BI), and gingival index (GI) of the two groups of patients decreased after treatment. After treatment, compared with the control group, the PLI, PD, BI, and GI of the research group decreased (*P* < 0.05). The total incidence of complications in the research group was (11.11%), and the total incidence of complications in the control group was (16.67%); there was no significant difference between the two groups (*P* > 0.05). After treatment, compared with the control group, the quality of life scores of the patients in the research group were reduced (*P* < 0.05).

**Conclusion:**

Root canal therapy and full crown restoration have a definite curative effect in patients with cracked teeth and chronic pulpitis, which can improve the inflammatory response, restore chewing function, maintain periodontal health, improve the quality of life, and do not increase the incidence of complications, so it has good application value.

## 1. Introduction

Because of caries, long-term wear of the tooth, and other factors, it will lead to high and steep cusp, increase cusp slope, weak tooth tissue, poor crack resistance, and excessive horizontal force on the tooth, resulting in small nonphysiological cracks on the surface of the crown, which is a cracked teeth [1]. Cracked teeth is a common dental disease in clinic, and its onset is hidden. The main symptoms of the patient are occlusal discomfort, severe pain, dull pain, and chewing pain, which bring great pain to the patient [2]. With the continuous development of cracked teeth, most of the cracks gradually deepen to the pulp, and because of various bacteria, such as actinomycete, into the pulp, the pulp is infected and then leads to chronic pulpitis [3]. If the patients with cracked teeth and chronic pulpitis are not effectively intervened in time, the aggravation of the disease may lead to pulp degeneration and necrosis, and then facial swelling, fever, alveolar bone infection, and other manifestations, which will seriously affect their chewing, eating, biting, and other daily tooth functions and appearance [4]. In recent years, with the change of people's life style and diet structure, the number of patients with cracked teeth and chronic pulpitis has gradually increasing, which seriously affects the quality of life of patients. Therefore, how to take scientific and reasonable measures to repair cracked teeth and chronic pulpitis is the focus of oral field.

At present, most of the patients with cracked teeth and chronic pulpitis are treated with root canal therapy in clinical practice. Through root canal preparation, disinfection, and filling, this technique can clean up the infection in the root canal, relieve the pressure stimulation, avoid reinfection in the root canal, and prevent the disease from developing to periapical periodontitis, and it has the advantages of fewer follow-up visits and short course of treatment, which has been widely recognized in clinic practice [5]. However, due to the cracked teeth and damaged pulp in patients with cracked teeth and chronic pulpitis, the hardness of the tooth decreases and the degree of force on the tooth changes, which has a certain impact on the chewing function of patients. Therefore, we think it is necessary to carry out full crown restoration after root canal treatment, so as to restore the daily life of patients. Full crown restoration covers the whole crown surface by metal, all-ceramic, and other materials, which essentially reduces the damage of tooth structure, can effectively prevent crown fracture, restore the adjacent relationship, repair the shape, function, and beauty of the defective tooth, and protect the integrity of tooth tissue, which is widely favored by patients and physicians [6].

To this end, this study observed the clinical effect of root canal therapy combined with full crown restoration in the treatment of cracked teeth and chronic pulpitis and discussed its influence on the level of inflammatory factors and chewing function, in order to provide reference for clinical treatment. The report is as follows.

## 2. Materials and Methods

### 2.1. Research Object

From May 2018 to June 2020, 87 patients with cracked teeth and chronic pulpitis in our hospital were selected, including 49 males and 38 females, aged from 30 to 61 years, with an average age of (43.55 ± 4.82) years. The patients were randomly divided into the control group and the research group by random number method. There were 42 cases in the control group, including 22 males and 20 females, aged from 33 to 61 years, with an average age of (43.93 ± 4.57) years. The course of disease ranged from 1 to 8 months, with an average course of (4.16 ± 1.02) months. The locations of teeth were reported as follows: 12 cases of maxillary first molars, 8 cases of maxillary second molars, 15 cases of mandibular first molars, and 7 cases of mandibular second molars. There were 45 cases in the research group, including 27 males and 18 females, aged from 30 to 59 years, with an average age of (43.20 ± 5.11) years. The course of disease ranged from 1 to 8 months, with an average course of (4.07 ± 1.13) months. The locations of teeth were reported as follows: 13 cases of maxillary first molars, 7 cases of maxillary second molars, 17 cases of mandibular first molars, and 8 cases of mandibular second molars. There were no significant difference in gender, age, course of disease, and location of teeth between the two groups (*P* > 0.05). This study had been approved by the medical ethics committee of our hospital. All selected patients were informed of the purpose, method, and possible risks of the study and signed an informed consent.

#### 2.1.1. Inclusion Criteria

There were clinical manifestations such as cold and hot stimulation pain and fixed-point bite pain. There were obvious cracks on the occlusal surface, and the cracks could be seen clearly after staining with iodine tincture. The affected tooth was a molar, and the patient complained of clinical symptoms, and X-ray examination results showed that it was pulpitis caused by cracked teeth. Root canal therapy was needed. There were no contraindications related to root canal therapy; severe bending of the root canal, calcification of the root canal, and obstruction of the root canal. Patients could cooperate with the treatment and receive regular follow-up.

#### 2.1.2. Exclusion Criteria

Exclusion criteria included acute suppurative pulpitis and dental caries. The results of X-ray examination showed the tooth root was longitudinally cracked. In addition to cracks, there were other serious defects in the teeth; severe periodontal disease; periapical periodontitis; abnormal loosening of teeth; and large shadow of the root tip. The tooth had been split, and the crown was separated. Moreover, severe organic diseases; mental disease; malignant tumor disease; women during pregnancy and lactation; and patients who dropped out during the study period were included.

### 2.2. Research Methods

#### 2.2.1. The Research Group Used Root Canal Therapy Combined with Full Crown Restoration

Preoperative assessment was performed before treatment, informed of the patient's own tooth condition, treatment procedures, and possible phenomena after treatment, and X-rays were taken to determine the direction and length of root canal of the teeth, whether the root tip had lesions and the degree of lesions. 4% articaine-epinephrine was used for local anesthesia. The pulp cavity was opened, the medullary cavity was cleaned, and humus was removed. ProTaper nickel-titanium root canal file was used for root canal preparation; try to avoid damaging the pulp bottom tissue. The root canal was enlarged with a root canal file. The root canal was prepared to size 25–30, and the working length and thickness were determined with a apex locator, it could prevent infectious substances from being brought into the apex, thereby reducing the occurrence of a series of strong postoperative reactions. The root canals were rinsed with 3% hydrogen peroxide solution and sodium chloride injection for many times and then dried with sterile cotton to disinfect the root canals and kept the cavities sterile and dry. Calcium hydroxide was injected to seal the canals, and cavitation was used to temporarily seal the canals. After 1-2 weeks, the root canal was filled and the temporary seal was removed under microscope. AH PLUS paste (Bilan, France) was used as filling agent. AH PLUS was mixed according to the ratio of 1 : 1. 1/3 of the main gutta percha tip was dipped in part of AH PLUS to fill the root canal. The working tip of the heat carrier was heated and pressed to a distance of 3–5 mm from the apical foramen; the heating was turned off and the pressure was maintained for 10 s. After complete cooling, reheat for 1 s, exit the heat carrier, scald off the upper part of the root canal gutta percha, press the apical gutta percha vertically, inject hot gutta percha in sections until the root canal was full, and remove the excess AH PLUS. When filling the root canal, it is necessary to make light action to avoid excessive pressure and deepen the crack. X-rays were taken to check the filling condition and root canal sealing condition. The following points should be paid attention to when performing root canal therapy: ① During root canal preparation, it is necessary to check whether the enlarged instrument has threads loose or 90° bend marks on the edge end to prevent the instrument from breaking during the operation. ② If there were many necrotic tissues in the root canal, it was necessary to rinse and clean the root canal thoroughly for several times, and the pressure should be controlled during the rinsed to avoid damaged the root canal and its surrounding tissues. ③ Before root canal filling, confirm that the root canal was trimmed into a cone shape, and a barrier had been formed at the narrowed root canal. One week later, if there was no abnormal appearance of the affected teeth; full crown restoration was started. Routinely prepare the teeth, use silica gel to make an impression, infuse the model with anhydrite, and make a porcelain full crown. After completing the crown restoration, instruct the patient to try it on, adjust the occlusion, and use the dual-curing resin adhesive to secure the teeth crown; the restoration of the full crown was completed. After treatment, anti-inflammatory drugs and analgesics could be given to patients to prevent postoperative pain, inform patients to be admitted to hospital for examination when discomfort occurred, and the patients were asked to review on time. The postoperative precautions were informed, avoid biting hard objects, pay attention to keeping the oral cavity clean, brush teeth in the morning and evening, rinse mouth after meals, do not smoke or drink, do not carry out strenuous exercise, and maintain a good eating style and rest habits. All patients were followed up for 6 months, and the effect was evaluated. All the above operations were performed by the same physician.

#### 2.2.2. The Control Group Only Used Root Canal Therapy

The operation steps of root canal therapy were the same as those of the research group, and the teeth were filled with light-curing composite resin. All the above operations were performed by the same physician.

### 2.3. Observation Index

#### 2.3.1. Efficacy Evaluation Criteria

6 months after treatment, the therapeutic effect of the two groups was evaluated. Effective: the patient had no discomfort, no pain, looseness, gum swelling, no surrounding tissue inflammation, normal chewing, and X-ray showed no shadow around the apex; improvement: the patient's symptoms were relieved, the pain and gingival swelling were improved, the inflammation of surrounding tissue was alleviated, the chewing function was improved, and the periapical shadow was reduced on X-ray; ineffective: the patient's symptoms remain unchanged, pain, gum swelling did not improve, the surrounding tissues still had inflammation, chewing discomfort, and the X-ray film showed that the periapical shadow did not change or even expand. Total effective rate = (effective + improvement)/total number of cases × 100%

#### 2.3.2. Inflammatory Factors

Before treatment and 7 days after treatment, 3 ml peripheral venous blood was collected in the early morning on an empty stomach, centrifuge at 3500 r/min for 6 min, separate the serum, supernatant was put into EP tube and stored in refrigerator at −80°C for standby. The enzyme-linked immunosorbent method was used to determine the serum interleukin-1*β* (IL-1*β*) and IL-6 levels, and the immunoturbidimetric method was used to determine the C-reactive protein (CRP) level.

#### 2.3.3. Chewing Function

Before treatment and 6 months after treatment, the occlusal force of teeth was measured by occlusal force tester. The molar was selected as the measuring point, repeat the measurement 10 times, and take the average value. Weighing method was used to measure chewing efficiency, the patients were instructed to chew 2 g peanuts for 20 times on each side, spit into the cup and rinse mouth repeatedly, and spit out the mouthwash at the same time. The chewables were collected and mixed with distilled water, and 200 number of screen mesh was used to sieve it; the unfiltered residue was weighed, and the ratio of weight change before and after chewing was regarded as chewing efficiency. The larger the value, the better the chewing efficiency.

#### 2.3.4. Periodontal Index

Before treatment and 6 months after treatment, a full-mouth periodontal examination was performed. Periodontal index: plaque index (PLI), probing depth (PD), gingival sulcus bleeding index (BI), and gingival index (GI) were measured at 6 sites on the mesial, median, and distal buccal and lingual surfaces of each tooth. The plaque display agent was used in PLI, and the patients gargled the plaque display agent for 2 minutes. The red attachment sites on the teeth were observed. The 0–3-point scoring method was used. The higher the score, the more deposits in the marginal gingival area and the more severe the plaque. PD measured the distance from gingival margin to the bottom of pocket or sulcus with periodontal probe. BI used 1–4-point scoring method. The higher the score, the greater the tendency to bleeding gums; GI used 0–3-point scoring method. The higher the score, the more serious the gingival inflammation, swelling, and edema. All measurements were performed by the same operator.

#### 2.3.5. Complications

The incidence of complications in the two groups within 6 months after treatment was recorded, including gingival swelling, inflammation of teeth, severe pain, malocclusion, difficulty chewing, and other problems.

#### 2.3.6. Quality of Life

6 months after treatment, oral health impact profile- (OHIP-) 14 scale was used to evaluate the quality of life of the patients. There were 14 items in 7 areas, including functional limitation, physical pain, psychological discomfort, physiological disorders, mental disorders, human communication disorders, and disability. 0–4-point scoring method was used, with a total score of 0–56 points. The lower the score, the better the quality of life.

### 2.4. Statistical Methods

SPSS22.0 software was used for analysis, measurement data conforming to normal distribution were expressed as mean ± standard deviation, and *t*-test was used for comparison between groups. Count data was expressed as a ratio, and the comparison between groups was performed by *χ*^2^ test. *P* < 0.05 indicated that the difference was statistically significant.

## 3. Results

### 3.1. Comparison of Clinical Efficacy between Two Groups of Patients

The total effective rate of the research group (97.78%) was better than the total effective rate of the control group (85.71%), and the difference was statistically significant (*P* < 0.05), as shown in Figure 1.

### 3.2. Comparison of Serum Inflammatory Factor Levels between the Two Groups of Patients

Compared with before treatment, the serum levels of IL-1*β*, IL-6, and CRP of the two groups of patients decreased after treatment. After treatment, compared with the control group, the serum levels of IL-1*β*, IL-6, and CRP in the research group decreased, and the difference was statistically significant (*P* < 0.05), as shown in Figure 2.

### 3.3. Comparison of Chewing Function between Two Groups of Patients

Compared with before treatment, the bite force of teeth and chewing efficiency of the two groups of patients increased after treatment. After treatment, compared with the control group, the bite force of teeth and chewing efficiency of the research group increased, and the difference was statistically significant (*P* < 0.05), as shown in Figure 3.

### 3.4. Comparison of Periodontal Index between Two Groups of Patients

Compared with before treatment, the PLI, PD, BI, and GI of the two groups of patients decreased after treatment. After treatment, compared with the control group, the PLI, PD, BI, and GI of the research group decreased, and the difference was statistically significant (*P* < 0.05), as shown in Figure 4.

### 3.5. Comparison of Complications between the Two Groups of Patients

The total incidence of complications in the research group was (11.11%), and the total incidence of complications in the control group was (16.67%). There was no significant difference between the two groups (*P* > 0.05), as shown in Figure 5.

### 3.6. Comparison of the Quality of Life between the Two Groups of Patients

After treatment, compared with the control group, the quality of life scores of the patients in the research group were reduced, and the difference was statistically significant (*P* < 0.05), as shown in Figure 6.

## 4. Discussion

With the improvement of living standards, people pay more and more attention to teeth. The causes of cracked teeth mainly include age, weak tooth structure, abnormal tooth physiological morphology, changes in adjacent relationship, weakened tooth tissue strength, and uneven distribution of bite force, which mostly occur in the middle-aged and elderly people over 40 years old [7]. Cracked teeth have the characteristics of concealment and gradualness. The cracks in the early stage of the disease are very thin and easy to be ignored. With the continuous development of cracked teeth, the cracks gradually increase and deepen to reach the dental pulp, resulting in bacterial infection of the dental pulp, the formation of hardened dentin, and then inflammatory occurs [8]. In some patients, the range of inflammation is expanded, the lesion is close to the apical foramen, and the toxins invade the dental pulp, which will lead to the occurrence of chronic pulpitis, causing pain, swelling, and other clinical manifestations. In severe cases, they may even lose their teeth, which greatly reduce the chewing function of patients and pose a serious threat to people's dental health [9]. It has been reported [10] that the maxillary molars always keep the passive impact state during the chewing movement. At the same time, the abrasion of the oblique ridge is more serious, which leads to the formation of the steeper oblique point. Therefore, the molars have a greater risk of cracked. Our hospital has rich clinical experience in the treatment of oral diseases. By selecting 87 patients' molars for research, our doctors summarize and share years of experience to provide reference for clinical treatment.

At present, the clinical application of root canal therapy technology has entered a mature stage and has a good therapeutic effect. Root canal therapy is a key treatment for pulpitis. It can effectively remove adverse irritation, clean up the source of infection in the root canal, prevent the spread of infection, and improve clinical symptoms by removing necrotic or gangrene substances in the root canal [11]. This technique is easy to operate. Through such measures as open the medullary cavity, removal of the pulp tissue, root canal cleaning, canal sealing, disinfection, filling, and other measures, the purpose of removing necrotic tissue is achieved, and the root canal is prepared into a cone-shaped space and tightly filled in a dry and sterile state. It can not only avoid bacterial infections, promote periapical healing, but also achieve the purpose of stabilizing the tooth root [12]. In addition, root canal filling is an important step in root canal therapy; root canal filling can tightly seal every gap in the root canal, which is helpful to prevent reinfection. AH PLUS is a kind of epoxy resin material, its thermal expansion coefficient is close to that of the tooth, and it has strong permeability, stable volume, and good fluidity, which is widely recognized in clinic [13]. However, after the patient's root canal treatment, although the affected teeth is fixed, but because the pulp tissue is removed and the pulp cannot be preserved, the resistance of the dental tissue decreases and the toughness is reduced, which affects the subsequent nutrient absorption of the tooth and easily causes tooth fracture and then affects the patient's oral health. After the repair, when the patient chews hard food for a long time, it will form a point-to-point contact with more concentrated stress, which is easy to cause complications such as difficulty in chewing and occlusal discomfort, and it is difficult to maintain a good long-term curative effect. Full crown restoration is a kind of dental restoration method that uses restorative materials to cover the crown and cemented with cement, which can prevent tooth fracture, restore the occlusal relationship of the teeth, and maintain the order of the dentition tidiness [14]. In clinical practice, casting full crowns or porcelain full crowns are often used for full crown restoration, but the teeth after casting full crowns have poor aesthetics, and it is easy to cause gingival bleeding, redness and swelling, and other complications [15]. Therefore, in this study, we used porcelain full crowns for patients with cracked teeth and chronic pulpitis, which has the characteristics of good strength and high recovery accuracy. In the process of root canal therapy and full crown restoration, root canal therapy can reduce the number of teeth contact with bacteria, prevents the growth of bacteria, and reduces the periodontal index; full crown restoration can effectively fix the teeth, avoid tooth chipping, reduce the stimulation of the teeth, and ensure the integrity of the teeth. The combined application of the two methods in patients with cracked teeth and chronic pulpitis can not only eliminate the lesions, but also restore the teeth, restore the basic functions of the dentition, improve the aesthetics of the appearance, and significantly improve the living standards of patients. We found that compared with the control group, the research group had a higher total effective rate, lower periodontal index and lower quality of life scores, and no difference in the total incidence of complications. The results suggested that, for patients with cracked teeth and chronic pulpitis, only giving root canal therapy has a certain therapeutic effect, but it cannot achieve the ideal effect. After using root canal therapy and full crown restoration, it is conducive to maintaining the periodontal health of patients, improving the quality of life, and does not increase the incidence of complications.

In this study, we used root canal therapy and full crown restoration to treat patients with cracked teeth and chronic pulpitis. After treatment, the patients' serum IL-1*β*, IL-6, CRP, and other inflammatory factors levels decreased, and the bite force and chewing efficiency were increased, which suggested that root canal therapy combined with full crown restoration can improve the inflammatory reaction and restore chewing function in patients with cracked teeth and chronic pulpitis. Studies have found [16] that chronic pulpitis can cause inflammatory reactions in host cells. During the inflammatory reaction, lipopolysaccharides in the cells of related pathogenic bacteria can produce a variety of inflammatory factors, which can damage the supporting tissues of the teeth. Inflammatory reaction is closely related to the occurrence and development of acute pulpitis. IL-1*β* is a common pro-inflammatory factor, which mainly occurs in the acute phase of inflammatory reaction and can reflect the inflammatory status of the body; IL-6 is a pleiotropic cytokine, which participates in the transmission of inflammatory response, and can promote the accumulation of inflammatory cells in periodontal tissue, and has a key role in the body's defense mechanism. CRP is an acute phase protein, and its level rises when the body is infected, which can be used as an important marker for clinical monitoring of pulpitis status [17]. Root canal therapy can timely remove necrotic tissue in the pulp cavity, tightly seal the root canal system, isolate the adverse stimulation to the periapical tissue, and eliminate the source of infection, which helps to promote the healing of periodontal tissue, relieve inflammatory symptoms, and prevent the further expansion of the scope of inflammation [18]. We filled the root canal after root canal cleaning. By placing AH PLUS paste in the root canal of patients, it can promote the expression of alkaline phosphatase gene of dental pulp cells and induce the differentiation of dental pulp cells and dentin cells, and it also can inhibit the reproduction of bacteria in the root canal, promote the reconstruction of the tissue around the periapical, and thereby alleviate the inflammatory response of dental pulp tissue. The application of full crown restoration can help to restore the shape and function of teeth, narrow the gap between the teeth, and reduce the microbial infection, so it can eliminate periodontal lesions, promote periodontal tissue repair, and reduce the secretion of inflammatory factors. In addition, studies have shown [19] that due to the growth of oral plaque in patients, the available area for chewing is reduced, which results in a significant reduction of chewing sensitivity of patients with irreversible pulpitis of molars. We found that the use of root canal therapy combined with full crown restoration for patients with cracked teeth and chronic pulpitis has the effect of reducing bacterial production, improving occlusal relationship, and restoring effective chewing area, which can make the teeth evenly stressed and improve chewing function. Compared with the root canal therapy alone, the treatment combined with full crown restoration can reduce the stimulation to teeth, prevent saliva and food from infiltrating into the pulp cavity, and lead to the further growth of bacteria, which is conducive to the recovery of cohesive relationships and occlusal relationships, full crown restoration has good strength, wear resistance, corrosion resistance, biocompatibility, and is not easy to deform, strong bending resistance, realistic appearance, stable color, and smooth surface, which plays a key role in the restoration of chewing function.

## 5. Conclusion

In summary, root canal therapy and full crown restoration have a definite curative effect in patients with cracked teeth and chronic pulpitis, which can improve the inflammatory response, restore chewing function, maintain periodontal health, improve the quality of life, and do not increase the incidence of complications, so it has good application value.

## Figures and Tables

**Figure 1:** Comparison of clinical efficacy between two groups of patients. Compared with the control group, ^*∗*^*P* < 0.05.

**Figure 2:** Comparison of serum inflammatory factor levels between the two groups of patients. Compared with the control group, ^*∗*^*P* < 0.05; compared with before treatment, ^#^*P* < 0.05.

**Figure 3:** Comparison of chewing function between two groups of patients. Compared with the control group, ^*∗*^*P* < 0.05; compared with before treatment, ^#^*P* < 0.05.

**Figure 4:** Comparison of periodontal index between two groups of patients. Compared with the control group, ^*∗*^*P* < 0.05; compared with before treatment, ^#^*P* < 0.05.

**Figure 5:** Comparison of complications between the two groups of patients.

**Figure 6:** Comparison of the quality of life between the two groups of patients. Compared with the control group, ^*∗*^*P* < 0.05.

## Data Availability

The data used during the study are available from the corresponding author upon request.
